# Functionalized Biomass Carbon-Based Adsorbent for Simultaneous Removal of Pb^2+^ and MB in Wastewater

This article has been retracted.

**DOI:** 10.3390/ma14133537

**Published:** 2021-06-25

**Authors:** Nannan Zhang, Nan Cheng, Qing Liu

**Affiliations:** 1 Modern Experiment Center, Harbin Normal University, Harbin 150025, China; 2 School of Chemical Engineering and Technology, Tianjin University, Tianjin 300350, China; Chengn1205@126.com

**Keywords:** adsorption, lignosulfonate sodium, complexation

## Abstract

It is of great significance to realize the sustainable development of the environment to synthesize functional materials by value-added utilization of waste resources. Herein, a composite material of polyacrylic acid/lignosulfonate sodium/cotton biochar (PAA/LS/BC) was successfully prepared by grafting polyacrylic acid with functionalized waste cotton biochar and lignosulfonate sodium. The obtained absorbent showed prominent capture ability toward Pb^2+^ and methylene blue (MB) with capture characteristics of the pseudo-second-order model and Langmuir isotherm model. This experiment explored the adsorption performance of the adsorbent for pollutants at different conditions, and further revealed the selective adsorption of Pb^2+^ and MB in the mixed system. Analysis confirmed that electrostatic attraction and complexation are the most critical methods to remove contaminants. Additionally, the regeneration and stability experiment showed that the adsorption capacity of PAA/LS/BC for pollutants did not significantly decrease after five runs of adsorption–desorption. Various results can demonstrate that the adsorbent has excellent performance for removing pollutants and can be used as a material with development potential in the field of adsorption.

## 1. Introduction

Environmental pollution has always been a major fatal problem that plagues mankind, among which water pollution is the most prominent problem. In a modern society with rapid industrial development, the discharge of wastewater caused by industrial production has become more and more serious, which has caused different levels of pollution in rivers and lakes [1,2]. Heavy metal ions and dyes in wastewater can enter the human body under the action of biological circulation and eventually pose a potential threat to human health. On the other hand, the growing need for clean water and the limited amount of water resources on Earth are forcing us to evolve our wastewater treatment [3,4,5].

Pb^2+^ is the most common toxic metal ion in daily life; whether it is a child or an adult, excessive intake of Pb^2+^ can cause irreversible damage to health [6]. Since 2009, there have been frequent incidents of Pb^2+^ poisoning among children; in August of the same year, 851 local children were poisoned by wastewater discharged from a local smelter in Fengxiang County, Shaanxi Province, China, with more than 170 children sent to hospital for emergency treatment, which caused riots among the local people and the government’s attention. Then, in 2011, waste from a battery factory in Huaining County, Anhui Province, caused excessive levels of Pb^2+^ in the blood of 228 children in the area, illustrating how dangerous heavy metal ions can be. Therefore, the treatment of heavy metal ions in wastewater is imminent [7]. The dyes in the wastewater can not only reduce the transparency of the water, but also consume a large amount of oxygen, which causes the water body to lack oxygen, affecting the growth of aquatic organisms and microorganisms and destroying the self-purification function of the aquatic system [8,9]. Among the common cationic dyes, methylene blue (MB) is considered to be the most representative pollutant, it is easily soluble in water or ethanol, and the aqueous solution is alkaline and toxic. Because MB is stable in nature and extremely difficult to degrade in aqueous solution, it is necessary to develop an excellent method for the targeted removal of MB [10,11]. Therefore, the treatment of pollutants in wastewater is a major challenge at present. Up to now, the adsorption method is considered to be the most widely used method in water pollution treatment technology with its unique advantages, which is not only high efficiency, but its simple operation, and the fact it can remove a variety of different types of pollutants such as heavy metal ions and dyes [12]. The most important step in using adsorption technology to treat wastewater is to prepare an environmentally friendly, low-cost, and highly effective adsorbent with excellent affinity for pollutants [13,14].

As a natural polymer, the structure of sodium lignosulfonate (LS) is rich in active groups such as sulfonic acid groups and hydroxyl groups that can complex with pollutants; moreover, it can be widely extracted from plants and is a good matrix for preparing hydrogels. In previous reports, LS has been widely used in the field of wastewater treatment [15]. Sun et al. successfully prepared sodium lignosulfonate modified graphene hydrogel, which realized the efficient removal of Cr^6+^ in the aqueous solution [16]. Mu et al. prepared a porous lignosulfonate/chitosan adsorbent that effectively reduced the concentration of Cu^2+^ and Co^2+^ in wastewater [17].

Biochar has been used as an adsorbent for many years, mainly due to its rich pore structure and large specific surface area, while the original biochar had a limited number of surface functional groups due to the inherent characteristics of its raw materials [18]. Therefore, it often exhibits shortcomings such as insufficient adsorption capacity. In order to overcome these deficiencies in performance, it is necessary to conduct further research and exploration on biochar adsorbents. According to research reports, modification of biochar or a composite with other functional materials are two important ways to improve the adsorption performance [19,20]. Zhang et al. prepared a novel polyacrylic acid grafted chitosan and biochar composite material for the efficient and selective adsorption of heavy metals [21]. Another foreign scholar, Choudhary et al., used modified biochar synthesized from cactus leaves as a renewable adsorbent to evaluate the adsorption performance of organic and inorganic pollutants such as malachite green, Cu^2+^, Ni^2+^ heavy metals, etc. [22].

High-efficiency, inexpensive, and simple preparation methods are the main features of future adsorption materials. It can be seen from the above analysis that carbon materials have a wide range of sources and low cost. Therefore, it is necessary to find more carbon materials that can be obtained in large quantities and can further enhance the adsorption performance. Similarly, a natural high polymer is the main material for the preparation of adsorbents. In the same way, it is key to be able to find a large number of natural high molecular polymers that contain a variety of effective active functional groups in continuous exploration. The carbon material and the natural polymer material are compounded to prepare an adsorbent with excellent performance, which can realize the efficient removal of pollutants in wastewater.

Based on the above discussion, waste cotton was used as a biochar source to compound LS to obtain an organic–inorganic composite adsorbent for the removal of heavy metal ions and dyes in a single system and binary system. In this strategy, after the cotton biochar (BC) was activated, it can be used as a supporting framework for composite materials, which is mainly due to the complex internal porous structure formed during the activation process and its affinity for most heavy metal ions, so the invention produces an efficient and stable adsorbent through two steps. First, LS is uniformly distributed on the surface of BC to form a mixture, and then the mixture is grafted onto the polyacrylic acid chain to form a complex hydrogel under the action of an initiator and crosslinker. The prepared composite hydrogel exhibited good adsorption affinity for heavy metal ions and dyes due to its long hydrophobic chain, strong intermolecular force, and abundant active functional groups.

## 2. Experimental

### 2.1. Chemicals and Materials

In these reagents, acrylic acid (AA), sodium lignosulfonate (LS), potassium persulfate (KPS), potassium hydroxide (KOH), sodium hydroxide (NaOH), hydrochloric acid (HCl), nitric acid (HNO_3_), lead nitrate (Pb(NO_3_)_2_), absolute ethanol, and methylene blue (MB) were all provided by Sinopharm Group Co. Ltd., (Sinopharm, Shanghai, China). N,N-methylenebisacrylamide (NMBA) was derived from Tianjin Kemeiou Chemical Reagent Co. Ltd., (Kemeiou, Tianjin, China). The reagents required for this experiment were all analytical grade. In addition, the waste cotton needed to prepare the biochar came from discarded quilts.

### 2.2. Preparation Method

Pretreatment of support frame: 2 g of natural waste cotton was evenly dispersed in 7 M KOH solution and ultrasonicated for 0.5 h to make the surface of the cotton fully contact with KOH. After the cotton/KOH mixture was left at room temperature for 24 h, the excess KOH solution was filtered out. Then, the waste cotton was dried at 65 °C for 24 h. The dried waste cotton was put into tube furnace and heated at 400 °C for 0.5 h, then, the temperature was ramped to 800 °C for 1 h at a heating rate of 5 °C min^−1^ to activate the combination. After cooling the waste cotton sample to room temperature, it was repeatedly washed with deionized water to remove the residual KOH until the pH was neutral, and dried at 80 °C for 24 h. Finally, the cotton carbon sample was put in 5 M HNO_3_ solution with magnetic stirring for 1 h and then oxidized overnight. After being washed to neutral, the sample was dried for 24 h at 65 °C.

Synthesis of the PAA/LS/BC: composite adsorbent: This can be divided into three main steps. First, 2.830 g KOH was fully dissolved in 5 mL water, and 5 mL AA was slowly added to the KOH solution in the ice water bath environment; after the mixed solution was cooled to room temperature, dry cotton biochar samples were added and fully stirred for even distribution in the solution. Then, the homogeneous mixture with dissolved LS was added to the above solution. Finally, the composites were obtained by a water bath for 1 h under the action of KPS and NMBA. The obtained hydrogel was washed several times with absolute ethanol, then broken into lumps and kept at 80 °C until completely dry. Scheme 1 shows the specific synthesis mechanism.

### 2.3. Characterization of PAA/LS/BC

The Fourier transform infrared (FTIR) spectra of the LS, BC, and PAA/LS/BC hydrogel samples in the wavenumber range of 500–4000 cm^−1^ were measured by a Nichole Nexus 470 spectrometer (Nicolet, Madison, WI, USA). The surface morphology analysis of the PAA/LS/BC hydrogel samples before and after the adsorption of Pb^2+^ and MB was via a the JSM-7800F scanning electron microscope (SEM) (JEOL, Tokyo, Japan). The thermal stability analysis of the samples was performed by a STA 449C integrated thermal analyzer (Netzsch, Selb, Germany) manufactured in Germany. The nano ZS90 zeta potential analyzer (Malvern, Malvern, UK) was used to determine the zeta potential of PAA/LS/BC at different pH.

### 2.4. Adsorption of Pb^2+^ and MB by PAA/LS/BC

All experiments were performed in 50 mL beaker. A sample of 0.01 g dry adsorbent was put into the test solution, and the concentration of the remaining pollutants in the supernatant after the adsorption equilibrium was reached was determined. The adsorption amount of PAA/LS/BC for Pb^2+^ and MB can be calculated by the following Equation (1):

(1) $$q_{e}=\frac{(C_{0}-C_{e})V}{m}$$

In this equation, *C*_0_ and *C_e_* (mg L^−1^) are the concentrations of pollutant at initial time and equilibrium time; *V* (mL) is the volume of solution; and *m* (g) represents the amount of adsorbent participating in the experiment.

### 2.5. Adsorption Experiments in Single System

All experiments were carried out at room temperature and the residual concentration of pollutants in the solution was determined at the time of adsorption equilibrium. To explore the effect of pH on adsorption, 0.01 g of the prepared PAA/LS/BC adsorbent was put in Pb^2+^ solution with pH 2–6 and MB solution with pH 2–12 for the adsorption experiments. The effect of the amount of adsorbent on the experimental capacity was completed by adding different doses of PAA/LS/BC (0.01–0.06 g). The kinetic study was carried out at a Pb^2+^ concentration of 50 mg L^−1^ and MB concentration of 25 mg L^−1^, the adsorption time of Pb^2+^ lasted for 3 h, and the supernatant was taken at different time intervals for measurement; similarly, the adsorption time for MB lasted for 24 h. The exploration of adsorption isotherms was carried out in pollutant solutions with different initial concentrations, the initial concentration of Pb^2+^ was 50–100 mg L^−1^, and the initial concentration of MB was 5–30 mg L^−1^.

### 2.6. Selective Adsorption

Simultaneous adsorption experiments of PAA/LS/BC on cationic dyes and metal ions were conducted to explore the competitive adsorption effects among the different pollutants. The adsorption experiment of Pb^2+^ with the initial concentration of 50–100 mg L^−1^ was carried out under the interference of MB (15 and 25 mg L^−1^) in the binary system of MB–Pb^2+^. In the same way, PAA/LS/BC adsorbed MB with a concentration of 5–30 mg L^−1^ in the presence of Pb^2+^ (15 and 25 mg L^−1^).

### 2.7. Reusability Test of PAA/LS/BC

The PAA/LS/BC adsorbent with Pb^2+^ and MB was completely desorbed with 0.1 M HCl, and then fully washed with deionized water for the next cycle of adsorption. Equation (2) is the adsorption cycle efficiency formula.

(2) $$\alpha =\frac{C_{0}-C_{e}}{C_{0}}\times 100\%$$

where α represents the cycle adsorption efficiency.

## 3. Results and Discussion

### 3.1. Characterization

#### 3.1.1. SEM

The surface morphology of PAA/LS/BC before and after the adsorption of Pb^2+^ and MB was determined. As shown in Figure 1A,B, there were many pores on the surface of the adsorbent, which is conducive to the combination of heavy metal ions and dyes with PAA/LS/BC. After the Pb^2+^ wase trapped by the adsorbent (Figure 1C), the pores disappeared and the surface became rough due to being covered by heavy metal ions. After MB was adsorbed (Figure 1D), the surface of PAA/LS/BC presented a completely different morphology, not only were there many tiny particles attached, but the surface also showed a layered stacking structure of irregular sheets [23]. This is because the adsorbed heavy metals existed in the form of ions in the solution and were mainly removed in the form of complex complexes formed by coordination reactions with the adsorbents. However, the physical and chemical properties of Pb^2+^ and MB were different, which led to the difference in the interaction between these two pollutants and the adsorbent, so that the adsorbent saturated with different pollutants showed a different surface morphology [24].

#### 3.1.2. FTIR

The infrared spectrum of each sample can be seen in Figure 2A. The characteristic peak of the–SO_3_H group belonging to LS was located at 1220 cm^−1^ clearly, and the peaks related to the asymmetric and symmetric stretching vibrations of the S=O group were found at 1113 cm^−1^ and 1040 cm^−1^. For BC, after activation and modification, the stretching vibration attributed to the typical carboxyl group of C=O was observed at 1700 cm^−1^, and there was a signal peak at 1100–1000 cm^−1^ belonging to the tensile vibration of C–OH [25]. In addition, both LS and BC had absorption peaks related to the bend vibration of O–H located at 3400~3500 cm^−1^ and stretching vibration peaks attributed to C–H around 2900 cm^−1^ [26]. In the FTIR of PAA/LS/BC, there were both LS and BC characteristic absorption peaks, not only that, due to the N–H stretching vibration of the amide, a new signal appeared at 1588 cm^−1^. All these results indicate that N, N-methylenebisacrylamide was used as the cross-linker to successfully synthesize the PAA/LS/BC composite [27].

#### 3.1.3. TGA (Thermogravimetric Analysis)

The thermal stability comparison of LS, BC, and PAA/LS/BC is shown in Figure 2B,C, in the range of 25–800 °C, and the total decomposition amounts of LS, BC, and PAA/LS/BC samples were 56.6 wt.%, 25.6 wt.%, and 53.1 wt.%, respectively. From the perspective of weightlessness, the weight loss of BC (25–800 °C) mainly came from physical adsorption or evaporation of structured water [28]. For LS, the slow drop in the range of 25–250 °C was attributed to the evaporation of adsorbed water, and the major weight loss from 250 to 800 °C resulted from the decomposition of backbone and the removal of oxygen-containing functional groups. For PAA/LS/BC, in addition to the initial moisture evaporation, the graft polymer chain scission and polymer pyrolysis movement were carried out at 250–410 °C; at 410 to 800 °C, the main chain of the polymerization gradually broke down until it was completely decomposed [29].

### 3.2. Effect of Solution pH and the Amount of PAA/LS/BC on Adsorption

The surface charge state of the adsorbent is a major factor restricting the adsorption capacity. Since Pb^2+^ exists in the form of divalent cations in the solution, which can precipitate to interfere with the experimental results at pH > 6, only the experiments with pH ≤ 6 were considered [30]. As presented in Figure 3A, the presence of excessive H^+^ in the solution hindered the adsorption of heavy metal ions by PAA/LS/BC at pH ≤ 3. As the pH increased, the adsorption amount of the adsorbent for Pb^2+^ gradually increased and tended to be stable, at this time, the electrostatic repulsion no longer affects the removal ability. For the adsorption of MB, it was also shown from the low adsorption amount at low pH to the enhancement of the adsorption amount at high pH [31]. These results can also be seen from the zeta potential (Figure 3B); when the pH < pH_zpc_ (zero charge point), the adsorbent surface is positively charged, and the electrostatic repulsion limits the removal of heavy metal ions and dyes by PAA/LS/BC. When pH > pH_zpc_, the adsorbent surface is negatively charged and the surface active site of the adsorbent is the key to determining the adsorption amount [32]. In summary, the removal of Pb^2+^ and MB by PAA/LS/BC was mainly accomplished by electrostatic attraction and surface complexation.

The amount of adsorbent directly determines the number of adsorption sites. As shown in Figure 3C, the adsorption amount of PAA/LS/BC to pollutants decreased continuously with the increase in the amount of adsorbent. In theory, the increase in the amount of adsorbent should promote the increase in adsorption amount [33]. Since the concentration of pollutants in the solution was constant, it is worth noting that a large number of adsorbents in the solution would agglomerate, which would result in some adsorption sites were not fully utilized. Therefore, the increase in the amount of adsorbent led to a decrease in the adsorption amount. In actual wastewater treatment applications, it is important to ensure that the adsorption efficiency is maximized [34].

### 3.3. Adsorption Kinetics

The adsorption amount of PAA/LS/BC to pollutants during the contact time can be seen in Figure 4A,B. Whether PAA/LS/BC adsorbs heavy metal ions or dyes, it is from the initial rapid adsorption to the final equilibrium stage. In the initial stage, a large number of adsorption sites on the surface of the adsorbent ensured the initial rapid adsorption, with the continuous interaction between the adsorbent and pollutants, the adsorption sites were constantly exhausted [35]. As a result, the adsorption reached equilibrium. Kinetic fitting was performed on the experimental data, and the two kinds of kinetic model equations are shown as follows:

Pseudo-first order model is shown in the following Equation (3):

(3) $$q_{t}=q_{e}(1-e^{-k_{1}t})$$

Pseudo-second order model is shown in the following Equation (4):

(4) $$q_{t}=\frac{k_{2}q_{e}{}^{2}t}{1+k_{2}q_{e}t}$$

In these two equations, the adsorption amount of PAA/LS/BC on Pb^2+^ and MB at equilibrium and time *t* are expressed by *q_e_* (mg g^−1^) and *q_t_* (mg g^−1^), respectively. The adsorption rate constants associated with the two kinetic models are *k*_1_, *k*_2_.

The relevant parameters obtained according to the kinetic model fitting diagram are listed in Table 1. Undoubtedly, the coefficient of determination (*R*^2^) of the pseudo-secondary kinetic model was closer to 1, which is consistent with the fitting curve. Additionally, the equilibrium adsorption value calculated by the pseudo-second-order kinetics could better reflect the development trend of the experiment. All of the above can show that the interaction between the heavy metal ion and the dye was chemical adsorption [36].

### 3.4. Adsorption Isotherms

In general, the effect of initial concentration on the amount of adsorption is explored by the relationship between the adsorbate and adsorbent. The isotherms curves for the removal of Pb^2+^ and MB by PAA/LS/BC are depicted in Figure 5A,B, where the removal ability of the adsorbent for these two pollutants was enhanced with the increase in the initial concentration of the pollutants until equilibrium [37]. This is mainly due to the large mass transfer driving force caused by the increase in concentration, which makes it easier for the contaminants to adhere to the adsorbent. In this regard, isotherm fitting was performed on the adsorption data, and the following are the three isotherm model equations used in this experiment.

Langmuir is shown in the following Equation (5):

(5) $$q_{e}=\frac{q_{m}K_{L}C_{e}}{1+K_{L}C_{e}}$$

Freundlich is shown in the following Equation (6):

(6) $$q_{e}=K_{F}C_{e}{}^{1/n}$$

Temkin is shown in the following Equation (7):

(7) $$q_{e}=A+B\ln C_{e}$$

where, the adsorption amount of PAA/LS/BC to Pb^2+^ and MB at equilibrium is expressed by *q_e_* (mg g^−^^1^), and *C_e_* (mg L^−^^1^) represents the residual concentration of pollutants in the solution at the adsorption equilibrium. Besides, *K_L_* is the Langmuir constant related to adsorption energy, and *n* and *K_F_* are both the Freundlich constant. *A* (mg L^−^^1^) and *B* are also constants about the Temkin model.

The relevant parameters obtained from the isotherm fitting of the experimental data are shown in Table 2. It can be clearly found that the coefficient of determination (*R*^2^) obtained according to the Langmuir model was closer to 1 than the other models. Therefore, it can be inferred that the adsorption behavior of PAA/LS/BC on Pb^2+^ and MB is the same adsorption mechanism, as both belong to the chemical adsorption on the monolayer [38].

### 3.5. Selective Adsorption

In terms of wastewater treatment in reality, there are many different types of pollutants in wastewater. On the basis of the above experiments, the selective adsorption of Pb^2+^ and MB by PAA/LS/BC in a binary system was also investigated [39,40].

In Figure 6A,B, it can be seen that in the Pb^2+^-MB system, despite the increasing concentration of Pb^2+^, the removal ability of PAA/LS/BC on MB remained stable basically with the interference of heavy metal ions that was due to the strong interaction between PAA/LS/BC and MB, which remained unaffected even in the presence of interference from other pollutants [41]. In contrast, in the MB-Pb^2+^ system, the removal ability of PAA/LS/BC on Pb^2+^ increased with the increase in MB concentration in the mixed solution. In this regard, the analysis of the experimental results showed that there are two different types of adsorption sites for the removal of Pb^2+^. It can be seen from the adsorption isotherm that the adsorption of pollutants by the adsorbent belongs to single-layer adsorption, whereas two layers of complex surfaces formed on the PAA/LS/BC when Pb^2+^ was adsorbed in the MB-Pb^2+^ system, which is called synergistic adsorption, where a previous study also found similar collaborative adsorption effects [42]. Not only does PAA/LS/BC provide active sites such as sulfonic acid groups and hydroxyl groups for the adsorption of Pb^2+^, but the -NH_2_ and -NH- groups on MB can also interact with Pb^2+^, where the cooperation of these two mechanisms together promoted the removal of Pb^2+^ by the adsorbent in the binary system.

### 3.6. Reusability of PAA/LS/BC

Good reusability is an important criterion to evaluate whether the adsorbent has a development prospect. In response to this, five adsorption–desorption experiments were carried out, and the results can be seen in Figure 7. The adsorption amount of PAA/LS/BC for Pb^2+^ and MB did not decrease significantly even after five cycles. It is normal for the adsorption amount to decrease slightly with each cycle because some of the contaminants do not completely detach from the adsorbent. In light of the good adsorption performance and reusability of PAA/LS/BC, it can be regarded as a kind of adsorbent with great potential.

### 3.7. Comparison with Other Removal Method

Table 3 shows the comparison between this method for removing Pb^2+^ and MB with other methods. It can be seen that there are various removal methods including ion exchange, chemical precipitation, biological adsorption, etc. First of all, surface complexation is chemical adsorption, which is stronger than biological adsorption and precipitation. Second, its selectivity is better than ion exchange, which can remove heavy metal ions and dyes at the same time. Third, other methods have requirements for the pH of the solution. Finally, from the removal results, the *q_e_* value of pollutants removed by the surface complex method used in this experiment was significantly higher than other methods. To sum up, it can be considered that the surface complexation used in this experiment is an excellent method to remove pollutants compared with other removal methods.

## 4. Conclusions

The preparation of PAA/LS/BC materials from waste cotton resources is a new approach to remove Pb^2+^ and MB in wastewater. For this experiment, the pseudo-second-order kinetics and Langmuir isotherm model indicate that the interaction between the synthesized adsorbent and Pb^2+^ and MB belongs to chemisorption on the monolayer. The removal amounts of Pb^2+^ and MB by PAA/LS/BC were 201.5 mg g^−1^ and 108.6 mg g^−1^ in the single system, respectively. It is interesting that the MB molecules present in the binary system promoted the absorption of Pb^2+^ by the adsorbent, while the adsorption amount of the adsorbent to MB remained stable in the adsorption environment with the co-existence of Pb^2+^. Finally, the good reusability enables the adsorbent to be reused. Taken together, this research is helpful to optimize the utilization of waste cotton resources to repair the aquatic environment polluted by heavy metal ions and dyes.

## Figures and Tables

**Scheme 1:** Synthetic mechanism of PAA/LS/BC.

**Figure 1:** SEM images of PAA/LS/BC (**A,B**), SEM images of PAA/LS/BC after adsorption of Pb^2+^ (**C**), and MB (**D**).

**Figure 2:** FTIR spectra of LS, BC, and PAA/LS/BC (**A**); TG (thermogravimetry) (**B**) and DTG (differential thermogravimetry) (**C**) curves of LS, BC, and PAA/LS/BC.

**Figure 3:** The effect of pH on PAA/LS/BC adsorption of Pb^2+^ and MB (**A**); the zeta potential of PAA/LS/BC at different pH (**B**); the effect of adsorbent dose on PAA/LS/BC adsorption of Pb^2+^ and MB (**C**).

**Figure 4:** Adsorption kinetics of Pb^2+^ and MB by PAA/LS/BC: pseudo-first-order kinetics (**A**) and pseudo-second-order kinetics (**B**).

**Figure 5:** Adsorption isotherms of Pb^2+^ (**A**) and MB (**B**) by PAA/LS/BC.

**Figure 6:** Adsorption amount of PAA/LS/BC to MB in Pb^2+^-MB system (**A**); adsorption amount of PAA/LS/BC to Pb^2+^ in MB-Pb^2+^system (**B**).

**Figure 7:** Reusability of PAA/LS/BC for Pb^2+^ and MB uptake in five runs of adsorption–desorption cycle.

**Table 1:** Kinetic constants of the adsorbents for Pb^2+^ and MB.

Type of Pollutant	Pb^2+^	MB
Pseudo-First-Order Model		
*q_e_* (mg g^−1^)	203.5	109.1
*k*_1_ (min^−1^)	0.031	0.248
*R* ^2^	0.988	0.933
Pseudo-Second-Order Model		
*q_e_* (mg g^−1^)	233.8	121.3
*k*_2_ (g mg−1 min^−1^)	1.5 × 10^−4^	0.003
*R* ^2^	0.994	0.998

**Table 2:** Isotherm parameters of the adsorbents for Pb^2+^ and MB.

Type of Pollutant	Pb^2+^	MB
Langmuir		
*q_m_* (mg g^−1^)	452.5	230.9
*K_L_* (L mg^−1^)	0.091	0.144
*R* ^2^	0.979	0.911
Freundlich		
*K_F_* (L g^−1^)	173.2	49.43
*1/n*	0.164	0.367
*R* ^2^	0.840	0.831
Temkin		
*A* (mg L^−1^)	191.3	12.21
*B*	43.82	50.24
*R* ^2^	0.884	0.904

**Table 3:** A comparison of the method for removing Pb^2+^ and MB with other reported methods.

Adsorbent	Removal Method	Adsorbate	pH	q_e_ (mg/g)	Ref
CPEMF	Chemical precipitation	Pb^2+^	8.5	Not given	[43]
BC400	Ion exchange	Pb^2+^	5 ± 0.05	57.13	[44]
CSMS	Biosorption/precipitation	Pb^2+^	3	125.2	[45]
WS-BC + BM	Ion exchange and precipitation	Pb^2+^	5.0	134.68	[40]
PAA/LS/BC	Coordination complex	Pb^2+^	6	201.5	This study
TC	Biosorption	MB	5	88.62	[46]
Ag@CdSe/Zeoilte	Catalytic degradation	MB	8	10.75	[47]
AC	Chemisorption	MB	7	24	[48]
OHC	Chemical interaction	MB	7	86.7	[49]
PAA/LS/BC	Coordination complex	MB	6	108.6	This study

## Data Availability

Exclude this statement.
